# A Study on *Glycyrrhiza glabra*-Fortified Bread: Predicted Glycemic Index and Bioactive Component

This article has been retracted.

**DOI:** 10.1155/2022/4669723

**Published:** 2022-08-30

**Authors:** M. Prabhahar, Gomathi K, Prakash S, Sendilvelan S, Saravana Kumar M, Jijina GO, Edwin Geo Varuvel, Haiter Lenin A

**Affiliations:** ^1^Department of Mechanical Engineering, Aarupadai Veedu Institute of Technology, Vinayaka Mission's Research Foundation, Deemed to be University, Chennai, Tamilnadu, India; ^2^Department of Biotechnology, Dr.M.G.R. Educational and Research Institute, Chennai, India; ^3^Department of Mechanical Engineering, Dr.M.G.R. Educational and Research Institute, Chennai, India; ^4^Department of Biomedical Engineering, Aarupadai Veedu Institute of Technology, Vinayaka Mission's Research Foundation, Deemed to be University, Chennai, Tamilnadu, India; ^5^Department of Mechanical Engineering, Faculty of Engineering and Natural Sciences, Istinye University, Istanbul, Turkey; ^6^Department of Mechanical Engineering, Wollo University, Kombolcha Institute of Technology, Kombolcha Post Box no. 208, Ethiopia

## Abstract

Bread is one of the highest-selling food products throughout the world. Lots of demand arose from the bread producers by the consumers to convert the traditional bread into functional food. In this study, normal bread was converted to functional herbal bread by infusing it with extracts of *Glycyrrhiza glabra*. The functional components of the *Glycyrrhiza glabra* were analyzed by liquid chromatography-mass spectroscopy (LCMS). The antioxidant study revealed that the extract has high antioxidant potency. The present study also investigated the antidiabetic potency of the extract. Bread is fortified with various percentages of *Glycyrrhiza glabra*, such as 2, 4, and 6. The fortified bread was analyzed for various sensory and taste parameters. Biochemical assays such as the in vitro digestibility test and glycaemic index suggest that fortified bread reduces the glycaemic index. From the study, it was inferred that 6% of infused bread was found to have high potency as a functional food when compared to 2 and 4%. From the above study, it was suggested that fortified bread reduces the glycaemic index and is best suited for diabetic people and diet watchers.

## 1. Introduction

Bread is simple food considered a staple food globally [1]. Though large people consume the bread, it is still considered junk food as it is mostly made of refined flour [2]. An enormous research study evidenced that food products made up of refined flour were one of the major reasons for diabetes mellitus, constipation, and other metabolic disorders [3]. Prolonged constipation is unavoidable among consumers of white bread as it does not have dietary fiber [4]. This leads to other serious complications such as irritable bowel syndrome, cancer, diabetes, and cardiovascular diseases [5].

Bread is a simple and cheap food consumed globally for ages and acts as a sign of heritage among the most popular ethnic human races [6]. Prevention and creation of awareness among the consumers about white bread are not possible as bread runs through their family among ages. Instead, converting traditional bread into functional food devoid of the hazardous effects of bread would be the better solution [7].

A lot of interest has been developed among consumers regarding the usage of functional foods [8]. Incorporating active functional food into our diet considerably decreases many metabolic risks [9]. The glycaemic index is also one factor that is gaining considerable attention among consumers, especially geriatrics and diabetic patients [10]. The food that manages to be a low glycaemic index with other health benefits would be the star of the food industry.

Fortification of bread with herbs started to trend globally [11]. The functional herbs infused in bread should enhance the flavor and nutritive value, decrease glycaemic index, and make it rich in antioxidants [12]. Here, in this study, we planned to increase the functional and biological effect of bread by infusing it with *Glycyrrhiza glabra*, which is rich in antioxidants and has antibacterial, antiviral, antipsychotic, enhances bowel movement, and has antidiabetic effects. *Glycyrrhiza* glabra itself is a natural noncarbohydrate sweetener with zero calories [13]. Bread fortified with *Glycyrrhiza* glabra will be analyzed for various sensory and taste parameters, release index, glycaemic index, antioxidant potency, and antidiabetic effects.

## 2. Methodology

### 2.1. Materials

*Glycyrrhiza glabra* (Athimathuram) was brought from the Siddha Medicine store, and dry yeast and wheat flour were bought at neighborhood stores.

### 2.2. *Glycyrrhiza glabra* Extract Preparation

The root of *Glycyrrhiza glabra* was washed, dried, and ground into a fine powder. To 300 grams of the powder, 100 ml of boiling water was added and kept for 30 minutes. After the incubation period, the extract was centrifuged for 15 mins at 3000 g. The recovered supernatant was used for *in vitro* activities.

### 2.3. Assessment of In Vitro Antioxidant Activity

Following the method described in [14], the aqueous extract's antioxidant activity was tested. Moreover, 0.1 mM of DPPH solution was prepared using 15 ml of ethanol. Various concentrations of *Glycyrrhiza glabra* extract were added to 100 *µ*l of DPPH. The mixture was mixed and left to stand for approximately 30 mins at room temperature. The absorbance at 517 nm was measured using a UV-Vis spectrophotometer. DPPH is in charge. The samples' concentrations were compared to those of gallic acid, a known standard. Calculations were made using the acquired triplicates.

### 2.4. HRBC Membrane Stabilization Assay

The methodology was done using the protocol mentioned in [15]. In total, 2 ml of blood was drawn and added to a tube containing EDTA. From the stock, 100 *μ*L of blood was added to the various concentrations of the *Glycyrrhiza glabra* aqueous extract. The mixture was then incubated at room temperature for 30 mins. Blood with distilled water acts as a control. The sample mixture was centrifuged at 3000 rpm for 10 mins. The supernatant was taken from each tube and was added to 96-well plates. The absorbance of 517 nm was measured using a UV-Vis spectrophotometer. The triplicates obtained were calculated.

### 2.5. HRLCMS Investigations

HRLCMS of *Glycyrrhiza glabra* was analyzed with Agilent 6200 series liquid chromatography system (SAIF IIT Mumbai). The solvent system consists of 95% water (Solvent A): 5% acetonitrile (Solvent B) with an applied gradient, where the flow rate is 0.2 ml/min and the column temperature is 25°C. Hypersil GOLD 3 microns of size 100 × 2.1 MM was used. The injection volume was set to 5 L with a run time of 30 minutes, and the sample ionization was done in both positive and negative modes utilizing the ESI interface [16].

#### 2.5.1. a-Amylase Inhibitory Assay

According to the method in [17], different concentrations of the extract were mixed with dimethyl sulfoxide solution. The *α*-amylase was attenuated in a pH 6.8 phosphate buffer. After incubation, a 1% starch solution was added to all of the reaction mixture tubes. After then, the combination was given a 15-minute incubation. After 15 mins of incubation, the reaction was halted by adding 1 ml of di-nitro salicylic acid reagent to the tubes, which were then placed in a water bath for 10 minutes to boil. After cooling the mixture, distilled water (10 mL) was added to each reaction mixture tube. Absorbance 540 nm was measured with a microplate reader. Acarbose acts as the positive control.

(Absorbance of control—absorbance of test sample)/(absorbance of control) *x* 100 is the percentage of inhibition.

#### 2.5.2. *a*-Glucosidase Inhibitory Analysis

The *α*-glucosidase inhibitory assay was estimated using protocol [18]. In total, 112 *μ*L of potassium phosphate buffer was used and the pH is adjusted to 6.8, 20 *μ*L of enzyme solution of concentration 1 unit/ml was added, and 8 *μ*L of the extract was mixed and incubated at the temperature of the room for approximately 15 minutes in a 96-well plate. p-NPG (20 *μ*L) was then added and incubated for additional 15 minutes at 37 C. The reaction was stopped using 80 *μ*L of Na2CO3 solution. The absorbance of 405 nm was measured and evaluated. For control, 8 *μ*L of DMSO was added instead of control as well as blank. Acarbose serves as the positive control.

Inhibitory activity (%) = [1-(OD sample—OD sample blank)/(ODcontrol-OD blank)] *x* 100.

### 2.6. Preparation of *Glycyrrhiza glabra*-Fortified Bread Sample

The ingredients were mixed until smooth and soft and left to rest for 15 minutes. The dough was then molded using a container (0.2 mm thick) to give a cylindrical shape to the loaf. After baking at 120°C for 45 minutes, the bread was ready. The bread loaves were allowed to cool after the baking process. The crust was separated from the crumb. The *Glycyrrhiza glabra* was added in different levels like 2%, 4%, and 6% to form *Glycyrrhiza glabra*-fortified bread sample for investigational studies. The bread was prepared using the following ingredients, as shown in Table 1.

### 2.7. Quantification of *Glycyrrhiza glabra*

#### 2.7.1. *Glycyrrhiza glabra* Extraction

The quantity of *Glycyrrhiza glabra* in bread is analyzed using crumb samples of the bread before its digestion. The crumbs were freeze-dried, homogenized into powder kind, and additionally sieved with the help of mesh for extraction. In a 15 ml tube, 0.5 g fine bread powder was weighed and combined with 8 ml methanol using a vortex. The tubes were then incubated in boiling water at around 60°C for 5 minutes. The tubes were then placed in an orbital shaker at 300 rpm for 10 mins. The liquid extract and the solid fraction were obtained through centrifugation at 3000 rpm for 5 mins using Thermo Fisher Scientific, a cooling centrifuge. The liquid extract obtained is used for GCMS analysis.

#### 2.7.2. GC-MS Investigation

The samples obtained from the extraction–centrifugation were analyzed using the instrument JEOL GCMATE II GC, which has a maximum resolution of 6000, and a maximum calibrated mass of about 1500 daltons. The instrument is used to analyze complex organic and biochemical mixtures. The compounds passing out from the spectra were collected while they exited the column, which is then known and quantified using the mass-to-charge ratio (m/z) [19].

### 2.8. In Vitro Digestibility Study

#### 2.8.1. In Vitro Digestion of Bread

Based on the modifications made in the protocol [20, 21] as described by [22], the in vitro digestibility of bread was studied. In this method, the quantity of *α*-amylase was changed in the absence of the secretion enzyme. Freshly baked bread portions were filtrated in a 2 mm sieve, and 5 grams were combined with the reaction mixture that contained 4 ml stimulated salivary fluid, 975 *μ*L of water, and 25 *μ*L of 0.3 M CaCl2. The combination was therefore vortexed for approximately 20 seconds before being incubated for 2 minutes using a magnetic stirrer. The mixture was then used for the gastric and intestinal phases. This phase is known as the oral phase.

Gastric phase: the samples from the oral phase were combined with pepsin (8 ml), which is prepared with the stimulated gastric fluid of concentration 2000 U/ml, followed by the addition of 5 *μ*L, 0.3 M CaCl2 solution, 0.65 ml 1 M HCl (pH 3), and 1.3 ml water. The mixture was then incubated with continuous stirring at 37°C for 2 hrs.

Intestinal phase: the samples of gastric digestion were mixed along with the reaction mixture prepared with stimulated intestinal fluids of 100 U/ml for the trypsin activity and 16 ml pancreatin (pH 7). The samples were placed in a shaker for 2 hrs at 37°C.

All the sample tubes of the phase (intestinal) were prepared for 7 digestion time points as follows: 0, 20, 40, 60, 80, 100, and 120 mins. All the samples were then centrifuged at 4°C for about 10 mins. Then, 4 ml of ethanol was added to each tube containing 1 ml of supernatant to terminate the reaction which is taking place. Then the samples were used for glucose analysis.

#### 2.8.2. Reducing Sugar Released

The resultant mixture collected from the intestinal phase is then transferred to the dialysis tube. The mixture was then dialyzed for 5 hrs, 37°C with PBS buffer. Then, 0.5 ml of the dialysate was taken every 10 mins. The reduced sugar was analyzed by adding 0.5 ml DNS reagent to dialyzed samples, which were dialyzed and boiled for about 10 mins. A spectrophotometer has been used to determine the absorbance @ 540 nm. Reduced sugar expressed was calculated in terms of GE, mg/ml.

#### 2.8.3. Sensory Analysis of Bread

A score card was used for sensory analysis based on the desirability and undesirability of bread. They are evaluated on the color, texture, taste, and quality characteristics such as the color of the crust, crumb, mouthfeel, and overall quality. The evaluation was done by giving the bread to panelists consisting of both genders aged 25–50 years. The score for each parameter was assigned as per the panelist's suggestion, which is analyzed with the maximum score. This is carried out using a seven-point hedonic grading scale, with one as very poor, two as poor, three as fair, four as satisfactory, five as good, six as very good, and seven as excellent [23].

### 2.9. Components with Bioactivity

#### 2.9.1. Total Phenolic Content Evaluation

This method has been studied by the revised procedure of [24]. The reaction mixture was made by mixing 1 ml of Folin–Ciocalteu reagent, 100 *μ*L of the sample, and 2 ml of 10% sodium carbonate and incubating it for 60 mins at 37°C. The absorbance at 765 nm was measured using a UV-Vis spectrophotometer. The total phenolic content was measured in milligrams of gallic acid equivalent/grams of sample and compared to the standard gallic acid value.

#### 2.9.2. Flavonoids Content Evaluation

Based on the protocol described [25], 0.9 ml of *Glycyrrhiza* glabra sample and 75 *μ*L of 5% of NaNO2 solution were mixed. After 5 minutes of incubation, 150 L of 10% AlCl3.6H2O was added to the contents. The contents were then incubated for another 5 minutes at room temperature. Then, using distilled water, 0.5 ml of 1 M NaOH was added to the volume of the combination, bringing the total amount to 2.5 ml. The mixture was forcefully mixed, and the absorbance was read using a UV-Vis spectrophotometer at 510 nm. The extracts were substituted with distilled water in the blanks. Total flavonoids were discovered, and their quantity was represented as catechin equivalents per Gram of extract.

#### 2.9.3. Total Amount of Starch (TS)

The protocol [26] calculates the overall starch content. In total, 50 mg of the sample was mixed with 6 ml of 2 M KOH and shaken for roughly half an hour at room temperature in the orbital shaker. Then 3 ml of 0.4 M sodium acetate buffer, pH 4.7, was prepared, and 60 L-amyloglucosidase (bought from Sigma-Aldrich) was added to it. The composition was then incubated in a water bath at 60°C for 45 minutes. Glucose has been determined using a glucose oxidase/peroxidase kit.

#### 2.9.4. Glycaemic Index (GI)

A modified protocol was used as described [26]. Then 100 ml of the extract was incubated in 10 mL of pH1 HCl–KCl solution that had been prepared and adjusted. A total of 5,200 L of pepsin solution was added, and the mixture was kept at 40°C for 1 hour under constant shaking. By mixing 200 *μ*L pancreatic *α*-amylase solution and incubating it at the temperature of the room for 45 minutes, the pH is increased. The addition of 70 *μ*L of Na2CO3 solution stopped the enzyme process. To dilute the samples, 25 ml of tris-maleate buffer was added to each. A total of 5 mL of pancreatic *α*-amylase solution was added to the mixture, which was then incubated at room temperature with continual shaking. At various time intervals, 1 ml of sample aliquots have been obtained and put in boiling water with continual shaking for roughly 5 minutes. The enzyme reaction that has occurred in the reaction mixture is inactivated by this technique. After that, the samples were chilled. Then 3 mL 0.4 M sodium acetate buffer and 60 mL amyloglucosidase were added to the aliquots once more. After adding the solutions, the samples were incubated for 45 minutes at 60°C by shaking. The volume was raised to 10 ml with distilled water when the incubation period ended, and the samples were centrifuged. Moreover, 0.1 ml of aliquot will be transferred to a glass tube for glucose measurement, which is analyzed using a glucose oxidase—peroxidase kit. The absorbance of the reagent at 510 nm was measured using a UV-Vis spectrophotometer. Utilizing SigmaPlot 10.0, the data are plotted; thus, the concentration over time graph was calculated. The glycaemic index of the samples was calculated using the following formula: pGI = 39.71 + 0.549 HI. The hydrolysis index is a proportion of total glucose released compared to the standard glucose released from 0 to 180 minutes [27].

#### 2.9.5. Analytical Statistics

The experiments have been carried out in three. Using SPSS 20.0, the one-way ANOVA test with Ducan's test has been used for analyzing values, showing *p* < 0.05, to evaluate the significance of the sample.

## 3. Results and Discussion

In the modern era, worldwide, people are more conscious of the influence of diet on their well-being. This leads them to look for more nutritious food with fewer calories and infused with bioactive ingredients. As an alternative to extra supplements such as tablets, society started to lean towards herbal infusions in the food. Functional foods provide a natural way to offer enough quantity of bioactive compounds. They are, thus, more functional, expedient, and likable to the consumers.

### 3.1. Evaluation of In Vitro Antioxidant Activity

Food products rich in antioxidants prevents various metabolic disorders. It also helps and maintains the proper digestion of food and prevents various metabolic ailments such as cancer, diabetes, and cardiovascular diseases [28, 29]. The DPPH radical scavenging activity results are (Figure 1) compared with those of gallic acid, standard the antioxidant. Low concentrations have higher radical scavenging activity. Based on the results obtained, 95% of radicals were scavenged at lower concentrations. So, we can conclude that the scavenging effects of *Glycyrrhiza glabra* extract on DPPH radicals were potent for antioxidant activity and can be effectively used as a supplement for food sources.

### 3.2. Evaluation of Antihemolytic Activity

Hemolysis assay shows that *Glycyrrhiza glabra* is nontoxic and can be used for further experimental studies. Various concentrations of the extract were used to analyze toxicity studies against human RBC cells [30]. The results showed that control cells treated with Triton-X 100 resulted in 100% lysis. The assay results showed that the *Glycyrrhiza glabra* extract does not possess any toxicity towards the human RBC cells, as shown in Figure 2.

### 3.3. HRLCMS

About 100 compounds were identified in the extract of *Glycyrrhiza glabra* by HRLCMS. Based on the properties like retention time, molecular formula, and database formula, the most prevailing compounds were identified, and the relative compounds were found to have many medicinal properties, such hesperitin (Figure 3(a)), isoliquiritigenin (Figure 3(b)), irigenin (Figure 3(c)), ketoprofen glucuronide (Figure 3(d)), berberine (Figure 3(e)), 7-hydroxy-2′-methoxyisoflavone (Figure 3(f)), Genkwanin (Figure 3(g)). The positive and negative ionizations are depicted (Figures 3(h) and 3(i)).

#### 3.3.1. *a*-Amylase Inhibitory Assay

The antidiabetic activity of *Glycyrrhiza glabra* exhibited the highest inhibition rate of about 80%, which was seen at 100 *μ*g/ml concentration, and the lowest inhibition rate of about 20% was seen at 10 *μ*g/ml concentration (Figure 4). Acarbose is used as a positive control. The result proved that the extract is dose-dependent and exhibits an increase in inhibitory activity compared to the amylase enzyme.

#### 3.3.2. *a*-Glucosidase Inhibitory Assay

*a*-Glucosidase plays a significant role in modulating PP hyperglycemia. The aqueous extract of *Glycyrrhiza glabra* was studied for the *a*-glucosidase inhibitory activities determined by using pNGP as substrate. The present data revealed that concentrations like 10, 25, and 50 *μ*g/ml showed <50%, but concentrations like 100 and 500 *μ*g/ml showed >50% of inhibitory activity, as shown in Figure 5.

### 3.4. Quantification

#### 3.4.1. GCMS

The GC/MS analysis was analyzed for both organic and biochemical mixtures. The name and the retention time (Figure 6) exhibit the various phytochemical constituents of *Glycyrrhiza glabra* through GC/MS analysis.

#### 3.4.2. Sensory Analysis

Sensory analysis of bread samples is shown in Table 2. The results were studied using a 7-point hedonic scale.

The *Glycyrrhiza glabra*-fortified bread sample is compared with the control of the regular bread (white bread) based on their color, odor, taste, and sweetness [31]. The global smell was less in bread that was prepared using *Glycyrrhiza glabra* when compared to normal white bread, but the aroma was different with a sweet smell, which was liked by the tasters. There is an increase in the flavor of *Glycyrrhiza glabra*-fortified bread when compared with the control due to the taste of the root, which could be more significant to the sensory attributes and overall acceptability of bread. The formulated fortified bread prepared using the above-said concentration was found to have a very good positive effect on consumers' overall acceptability, even more among diabetes patients.

The parenthesis values indicate the maximum rating on the scorecard.  Figure 7 shows the radar plot for sensory evaluation of the board.

### 3.5. Bioactive Components

A lot of interest was raised among the consumers that the food they consume should satisfy the daily need for antioxidants [32].

Based on the biofunctional properties developed at the time of evaluation are analyzed at the retention time of the process. Total phenolic and flavonoids in the bread sample of *Glycyrrhiza glabra* showed an effective level of both phenolic content and flavonoids. From the analysis, it was found that in a dose-dependent manner, the total phenolics and flavonoids increased in the fortified bread. This shows that not only in taste but also functionally, the fortified bread shows more potency than the normal bread available in the market.  Table 3 shows the bioactive components of white bread and *Glycyrrhiza glabra*-fortified bread.

### 3.6. In Vitro Digestability Study

#### 3.6.1. In Vitro Digestion of Bread and Glycaemic Index

According to Figure 8, the in vitro digestion of bread shows dose-dependent inhibition of *Glycyrrhiza glabra* at the time of the release of reduced sugar. The gastric chyme transit through the whole small intestine will take about 4-5 hrs [33]. At 60 mins of dialysate, the concentration of resistant starch of sample bread with *Glycyrrhiza glabra* showed to be less when compared with the control sample. At the end of 240 mins of dialysis, the concentrations of resistant starch for *Glycyrrhiza glabra*-fortified bread samples at 2%, 4%, and 6% were reduced in a dose-dependent manner.

#### 3.6.2. Total Starch and Glycaemic Index

Based on the sensory evaluations, 6% *Glycyrrhiza glabra* extract was used for the in vitro starch digestibility studies. The levels of total starch, resistant starch, and digestible starch of the fortified bread products are shown in Table 4. Resistant starch ranges are about 3.99 ± 1.24. The *Glycyrrhiza glabra*-fortified bread exhibited higher values in resistant starch, resulting in lower digest ability starch. The prepared bread showed similar starch content to that in the normal bread. But the digestibility of the starch is found to vary. These kinds of variations are due to the protein and dietary fiber content. Based on the report in [34], when compared to other starches, wheat starch swells slowly. This is because the protein present around the starch granules stops the granule swelling and gelatinization of starch by reducing the enzymatic attack. Based on all these, the bread produced by the extract *Glycyrrhiza glabra* is rich in protein and dietary fiber. Therefore, they show increased levels of resistant starch with a rise in the extract concentration.

The hydrolysis index (HI) is calculated as the rate of hydrolysis over time (Figure 9) with the predicted glycaemic index (pGI), as shown in Table 4. Normal white bread shows a higher hydrolysis index and pGI, resulting in 48.00 ± 1.08 and 63.02 ± 1.47. *Glycyrrhiza glabra*-fortified bread samples showed less percentage of hydrolysis index and pGI, which ranged from 43.35 ± 1.20 to 22.16 ± 1.62 and 59.14 ± 0.99 to 52.15 ± 1.12. Jenkins et al., 2008, reported that food is organized into three stages: low (<55), medium (56–69), and high >70. The results show the extract has a low pGI and high-resistance starch. This further confirms that the biofunctional components will act effectively and inhibit the enzyme at postprandial hypoglycemia [35]. The therapeutic value of low GI in the food of diabetic patients is efficient. The low GI and highly resistant starch reduce insulin resistance by reducing the glucose levels in the blood of diabetic patients. It even improves lipid metabolism to prevent cardiovascular diseases.

#### 3.6.3. Quality Evaluation of Bread

The life of bread depends on the moisture content of the bread. The moisture content of bread made with extract *Glycyrrhiza glabra* is found to be high when compared to the normal bread we use. To maintain the quality of bread, the moisture content plays an important role, and these have an adverse effect on its preservation. Except for the sugar content, there is not much change in the proximity composition of the bread as we added only the extract that has a sweet taste with zero calories. The large difference in carbohydrate content of white bread and fortified bread is due to the complete avoidance of sugar while preparing the fortified bread. As the extract itself gives natural noncalorific sweetener, there was no need for the addition of sugar. This majority reduced the carbohydrate contents.  Table 5 shows the evaluation of the proximity composition of bread.

This study reveals that the infusion of *Glycyrrhiza glabra* extract did not change the traditional taste of the bread. Adding *Glycyrrhiza* glabra extract gives the natural sweetness to the bread without adding sugar to the dough. The noncarbohydrate sweetener also reduces the overall calories of the bread. Due to this, when compared to the normal bread available in the market, *Glycyrrhiza glabra* extract added bread was healthier with fewer calories. Due to this, diet watchers can make this bread their staple food without any hesitation. Moreover, this bread will be more suitable for diabetic patients due to its low sugar content and fewer calories. Also, the active ingredients in *Glycyrrhiza glabra* help to control the glycaemic index. This bread is an appropriate product to be used as a functional food as it satisfies the varied needs of the consumers.

## 4. Conclusion

This study shows that incorporating the extract of *Glycyrrhiza glabra* into bread completely avoids the usage of sugar. The total phenolic compound and antioxidant potency of the bread increased after being infused with the extract. The sweetness that arose from adding the extract was completely with zero calories. Apart from that, it was also found that the extract reduced the RDS, SDS, and RS and lowered the glycaemic index. It even shows that *Glycyrrhiza glabra* has the potential to be used in bakery products that have lots of health supplements. The bioactive components of bread, such as phenolics and flavonoids, are found to be increased in the Glycrrhiza glabra-fortified bread sample. Type 2 diabetes is caused by the participation of carbohydrate hydrolyzing enzyme in postprandial hypoglycemia. The overall findings in vitro of the fortified bread sample give us a potential result that this bread sample is suitable and recommended for diabetic patients due to the lower glycaemic effect of the *Glycyrrhiza glabra* in the preparation of bread.

## Figures and Tables

**Figure 1:** Antioxidant activity of *Glycyrrhiza glabra* extract.

**Figure 2:** Antihemolytic activity of *Glycyrrhiza glabra* extract.

**Figure 3:** (a) Hesperetin spectrum, (b) isoliquiritigenin, (c) irigenin, (d) keto glucuronide, (e) berberine, (f) 7-hydroxy-2′-methoxyisoflavone, (g) genkwanin, (h) positively ionized peaks of *Glycyrrhiza glabra* extract, and (i) negatively ionized peaks of *Glycyrrhiza glabra* extract.

**Figure 4:** Alpha amylase inhibitory assay of *Glycrrhiza glabra* extract.

**Figure 5:** *α*-Glucosidase inhibitory assay of *Glycyrrhiza glabra* extract.

**Figure 6:** GCMS graph of the *Glycyrrhiza glabra* extract.

**Figure 7:** Radar plot for sensory evaluation.

**Figure 8:** *Glycyrrhiza glabra* digestion trajectories.

**Figure 9:** Starch hydrolysis in *Glycyrrhiza glabra*-fortified bread.

**Table 1:** The recipe for 2%, 4%, and 6% *Glycyrrhiza glabra*-fortified bread.

Ingredients	Quantity	Quantity	Quantity
Wheat flour	300 grams	300 grams	300 grams
*Glycyrrhiza glabra* extract	2 g in 100 ml	4 g in 100 ml	6 g in100 ml
Yeast	7 grams	7 grams	7 grams
Salt	1%	1%	1%

**Table 2:** Sensory Comparison of normal white bread and *Glycyrrhiza glabra*-fortified bread.

*Glycyrrhiza glabra -*fortified bread	Color	Odor	Taste	Sweetness	Overall acceptability
(2%)	6	5	4	5	5
(4%)	6	6	6	5	5.8
(6%)	6	6	6	6.5	6.1
Normal white bread (control)	6	2	3	5	4

**Table 3:** Bioactive components of white bread and *Glycyrrhiza glabra*-fortified bread.

Bread samples:*Glycyrrhiza glabra-*fortified bread	Phenolic content mgGAE/100 g	FlavonoidsmgCE/100g
2%	66.76 ± 1.22	22.71 ± 0.68
4%	90.05 ± 1.19	25.54 ± 1.22
6%	103.02 ± 1.04	37.22 ± 1.33

**Table 4:** Starch digestibility and predicted glycaemic index of *Glycyrrhiza glabra*-fortified bread.

Bread sample: *Glycyrrhiza glabra-*fortified bread	Resistant starch%	Hydrolysis index%	Predictedglycaemicindex%
2%	4.86 ± 1.39	43.35 ± 1.20	59.14 ± 0.99
4%	6.04 ± 1.79	32.29 ± 2.19	46.19 ± 1.66
6%	11.57 ± 1.24	22.16 ± 1.62	36.15 ± 1.12
Normal white bread (control)	3.99 ± 1.24	48.00 ± 1.08	63.02 ± 1.47

**Table 5:** Evaluation of proximity composition of bread.

Bread sample	Moisture content %	Crude protein %	Crude fiber %	Ash content %	Lipid content %	Carbohydrate %	Crude fat %
Normal white bread (control)	16.1 ± 0.01	13.12 ± 0.01	2.45 ± 0.01	4.44 ± 0.68	3.77 ± 0.55	83.24 ± 0.01	3.38 ± 0.12
*Glycyrrhiza glabra-*fortified bread	17.8 ± 0.01	13.40 ± 0.68	2.57 ± 0.02	2.84 ± 0.01	3.09 ± 0.08	42.11 ± 0.58	3.30 ± 0.01

## Data Availability

No data were used to support this study.
